# Application and Feasibility Study of Integrated Nursing Information Construction in Nephrology Nursing

**DOI:** 10.1155/2022/7033840

**Published:** 2022-01-15

**Authors:** Liyan Jiang, Qiaoling Xie, Lingwei Chen

**Affiliations:** The First People's Hospital of Wenling, Wenling 317500, China

## Abstract

With the continuous deepening of medical reforms and the continuous attempts and explorations of various management models, the traditional health care model is undergoing tremendous changes, and patients' needs for medical institutions are becoming more and more comprehensive. Medical institutions are meeting the needs of providing medical services to patients at the same time. It is even more necessary to change our thinking and enhance the service concept. This article is based on case-based deep learning hospital nursing business process reengineering and the application and feasibility study of integrated nursing information construction in nephrology nursing. This article uses the literature analysis method, the social survey method, and other methods to discuss the construction of integrated nursing information. On the one hand, the content of this article uses the concept of process reengineering to analyze the current development status and existing problems of the hospital care industry and find countermeasures to solve problems. On the other hand, the main research content of this article is the construction of integrated nursing information and its analysis of the application and feasibility of nursing in the nephrology department. At the same time, under the background of the rapid development of the mobile Internet, we will carry out extended thinking on the continuous transformation of the construction of nursing information. According to the survey results, 87.5% of patients in the nephrology department are dissatisfied with the current hospital's work efficiency, and 85.7% of the nursing staff in the nephrology department are generally satisfied with the information management of the current department. After the implementation of the hospital information integration system, patient satisfaction is as high as 98.2%, and the satisfaction of medical staff reached 94.2%. The construction of integrated nursing information has played a great role in the application of nephrology nursing.

## 1. Introduction

Under the background of information integration, with the rapid development of computer technology, network technology, and communication technology, information construction has become a hot spot of concern to the whole society. The popularization of the Internet has provided unprecedented opportunities for the development of information technology. While the field brings opportunities, it also intensifies competition. The essence of the integrated construction of nursing information is that many medical systems are integrated horizontally, and data and information are seamlessly linked, so that hospitals, departments, and positions can be interconnected, breaking the traditional medical mode of vertical and gradual information transmission mode [1]. Information is the basis for the implementation of integrated and joint medical treatment.

With the continuous development and progress of society and the reform of the medical system, many experts and scholars began to discuss “how to continuously improve the level of medical care” [2]. This inevitably requires the hospital to make a comprehensive and thorough service process change. By building an integrated nursing information platform, all relevant information is entered into a unified interface, and the nursing manager provides basic patient information such as medical records and nursing cost-related information. It also helps to conduct organic integration and analysis. Based on the internal data of the system, a brand-new business process is designed to provide patients with a convenient and unobstructed medical environment. Therefore, how to improve the efficiency and quality of outpatient services, change the mode of outpatient services, and thereby improve patient satisfaction and hospital management performance has become a research topic for many scholars.

In recent years, as the informatization has gradually penetrated our daily lives, it has brought us convenience in various fields. All regions are exploring how to use informatization and processes to better provide patients with convenient and effective medical services. The Zhu and Gu study examined the impact of the comprehensive nursing handover system (structured content, minimal data set, and electronic modules in the patient clinical information system) on nurses' satisfaction with handover and practice changes [3]. Background: poor transmission of patient information between clinicians during handover is associated with poor patient outcomes. Design: evaluation method before and after using a hybrid method. Method: integrated care transfer system was introduced and evaluated in Australian hospitals. The revised Bradley clinical handover survey (*n* = 40 before and after *n* = 80) was used to measure changes in nurse satisfaction. Whalen et al. believes that when nursing and nursing services are integrated, real-time pickup and agency tasks also increase, which may lead to an increase in database queries, thereby increasing the amount of information transmitted [4]. In order to effectively solve this low-efficiency problem, his research aims to develop a nursing and nursing comprehensive information system that eliminates database queries and adopts real-time transmission of pickup and action information. Due to the increased workload and responsibilities of the new system, the ward agent dashboard has been developed so that each ward employee can grasp all the patients' behaviors in real time and improve the quality of service. Ghanadbashi and Ramsin believes that the current nursing management information system is a software system for processing nursing information established using information science theories and computer technology methods, and it is an important part of [5]. It can improve the utilization of important resources and the quality and efficiency of nursing work. Based on this, his article developed and applied the comprehensive management information system of obstetrics and gynecology and completed the analysis, design, and implementation of the system under the guidance of modern software engineering methods. These studies are of great value to the medical and health undertakings of today's society. All researchers are aware of the importance of the combination of current medical undertakings and informatization to expand the scope of services and improve the service structure. However, their research does all exist. Limitations are too focused on discussing a subtle point that the content of the research is not consistent with the main purpose of the article.

The integrated construction of nursing information relies on the development of informatization, intelligence, and platformization. The information platform is used to reengineer the conventional traditional business processes effectively and thoroughly, accompanied by the third characteristic of informatization and intelligent technology [6]. The continuous deepening of the subindustrial revolution has become the propeller for the formation, development, maturity, and gradual entry of the business process reengineering theory into practice. In order to adapt to the rapid development of society and science and technology, as well as the growing health needs and social needs in the development of the hospital nursing industry, this article is based on the use of case-based deep learning hospital nursing business process reengineering and the construction of integrated nursing information in nephrology nursing. The feasibility study carried out extensive research on the breadth and depth, based on the operation process and system testing of the business system of the nursing information platform, and carried out research on the integration of nursing information for nursing staff and patients in the department of nephrology. The impact on its application prospects is studied in [7].

## 2. Integrated Analysis of Nursing Information

### 2.1. Patients' Satisfaction with Nursing Work in the Nephrology Department

With the continuous promotion of the concept of “high-quality nursing service” throughout the country and related research and development, the concept of “consolidating basic nursing and providing satisfactory services” has been continuously deepened and developed in the nursing work of nurses. Nurses continue to improve themselves and perform their duties as nurses. Patients provide effective, high-quality, and satisfactory nursing services. Patient satisfaction has been included in the evaluation process of hospital standardization construction and has become an important index for evaluating hospitals [8]. As an important part of patient satisfaction, nurse service satisfaction affects overall hospital service satisfaction to a large extent. Patient satisfaction has become an important indicator for evaluating the quality of hospital medical services and analyzing key factors affecting patient satisfaction. Taking targeted measures to meet the health needs of different groups of people is of great significance to improving the quality of hospital services. In the original hospitals, the only way for doctors to obtain patient information was to visit patients in the ward, check some cases, or go to the nurse station by phone to find the head nurse to ask about the patient's condition [9]. Nurses need to keep a paper record of the collected physical data and case information, and then copy the information repeatedly. This processing method not only wastes cost, time, and manpower but also makes mistakes due to repeated copying of data, which affects the correctness and accuracy of data information. This not only shows that there are general problems in the current medical development, as the indispensable nurses and patients in the whole medical process, they cannot receive satisfactory care, which in turn affects the evaluation of patients' impression of the entire hospital [10].

### 2.2. Nursing Business Process Reengineering Theory

With the reform of the medical system and the state's repositioning of the nature of hospitals, competition in the medical industry has become increasingly fierce. Affected by the external environment, the competition among major hospitals has changed from a single factor to a comprehensive factor. Therefore, hospitals must use medical resources scientifically and rationally, and think and solve problems from the perspective of patients, to effectively enhance their competitiveness. The nursing work flow is based on an in-depth understanding and scientific analysis of the main business processes of the organization and is guided by customer needs. Effective planning, reorganization, or modification of the main business processes is carried out to improve the links in the business process to improve the quality of the entire operation, with the purpose of improving labor efficiency and reducing the overall cost of operations [11]. In short, it takes the process-oriented and core to thoroughly reshape the basic operation links to achieve significant results. Since the 1990s, foreign hospitals have been exposed to the theory of process management and started large-scale practical activities. Many medical institutions formulate different process reengineering programs according to the needs of patients and market competition and establish a patient-centric process organization to achieve the purpose of improving management models and improving management performance. The reengineering of hospital nursing business processes generally goes through four steps of needs analysis, planning, action, and monitoring [12].

Entering the hospital's information system through the patient's personal information makes the system state from *x* to *x* + 1. This process requires analysis [13]; when the patient is cured and discharged from the hospital, subsequent leaving of the system makes the system state from *x* to *x* − 1. The first process is the end of the needs analysis. The admission procedure to the discharge procedure is a system, and the general state of the system can be expressed as follows:

(1) $$\begin{array}{c} R_{T_{x}}=m\left(T_{x+1},T_{P_{x}}\right),\\ \left(x+1\right)mP_{x+1}+\gamma P_{x-1}=\left(\gamma +xm\right)P_{x},\;1\leq x<m, \end{array}$$

where *T*_*x*_ represents the time distribution of the arrival of customers during the input process, *T*_*p*_ represents the time distribution of the patient's stay in the hospital or the patient's information in the hospital system, and *R* represents the information system capacity [14]. When a certain patient is receiving nursing business, the business demand analysis in the hospital information system that is occupied is as follows:

(2) $$\begin{array}{c} Q_{x}=F\frac{1}{p}\sum_{x=1}^{t}R_{n-1},\\ R_{n}=\frac{1}{n}\left(\sum_{p}^{1}x_{n}-1\right), \end{array}$$

where *R*_*n*−1_ represents the overall information capacity after excluding the nth patient's remaining capacity [15].

Because there is the possibility of another patient's information output at the same time as the patient's information is entered, in order to ensure the effective reintegration or redesign of the overall hospital care business in this situation, we choose to use genetic algorithms to select, cross, and cross over. Mutation and other operations are adjusted to ensure accurate data update. The method of data integration of the genetic algorithm in nursing business process is [16] as follows:

(3) $$\begin{array}{c} R_{0}=\left\{\sum_{T_{1}}^{N}r+\frac{n_{m}}{P}\left(\lambda ,T_{0}\right)a\right\},\\ \frac{n}{\lambda }=\left(m,p\right)\sqrt[{2}]{T_{1}}a\frac{r}{N}, \end{array}$$

where *r* represents the total nursing business demand after the system is updated [17], and (*λ*, *T*_0_) represents the demand status when different patients end business services and start new nursing services. The data is sorted by the genetic algorithm, which can be efficiently arranged for process reengineering after monitoring the data. Process reengineering is just the beginning. Continuous improvement is the core of maintaining process reengineering.

### 2.3. Reliability Analysis of Integrated Nursing Information Construction

Since the mid-1990s, a large-scale hospital information integration system has been continuously developed in China, which incorporates nursing work such as ward bed data management, doctor order data statistics, and related cost settlement, which improves the efficiency of paper-based nursing work. But at present, there is a lack of nursing informatization talents in China, and there is a lack of unified standards related to nursing information systems [18]. So far, there is no special organization in the country to conduct research on hospital nursing information management standards, and the state and administrative departments have no unified plan for this. Plan the required data sources and data definitions. Through the organic combination of the data exchange platform and various information systems, the automatic extraction and conversion of data between the same database and different data formats at the customer's access terminal can be realized, and the heterogeneous distributed application system can quickly realize data integration between them. The reliability analysis of integrated nursing information construction can not only measure the reliability of system informatization in advance but also improve the weak links of the system and improve the reliability of the system [19]. In this regard, the reliability mathematical model method is used to verify the value of the integrated construction of nursing information.

As an object-oriented high-level programming language, C# has outstanding features such as simplicity, elegance, security, and stability [20]. It not only has the powerful functions of C and C++ at the same time, but also simplifies or directly subtracts a lot of complex features. In the construction of information management systems, recursive methods are often used, which are as follows:

(4) $$\begin{array}{c} D_{o}=1+\left\{1,2,3,\ldots ,x\right\}\left(S_{x\cdot \left(x-1\right)}\right), \end{array}$$

(5) $$\begin{array}{c} D_{x}=2D_{x-1}+1,\;\left(x>1\right). \end{array}$$

Equation (5) is a typical recursive formula [21]. If *S*_*x*_=*D*_*x*−1_+1, then *D*_*x*_=2*S*_*x*−1_ (*x* > 0), the solution of the recursive formula is as follows:

(6) $$\begin{array}{c} S_{x}=2^{x}. \end{array}$$

Thus, the following is obtained:

(7) $$\begin{array}{c} D_{x}=2^{x}-1,\\ D_{x}=\sum_{x=1}^{s}\frac{1}{3}\lambda \left(S_{x+1}\cdot x_{s-1}\right). \end{array}$$

It is very convenient to build an integrated nursing information system program with a high-efficiency development program, operation efficiency, and operational functionality [22]. Analyzing the reliability of the integrated construction of nursing information generally combines the relationships between various fields, such as parallel and hybrid. The parallel system is composed of multiple subdomain systems in parallel or redundant [23]. The reliability of the parallel system and the hybrid system can be expressed as follows:

(8) $$\begin{array}{c} S_{i}=1-\int_{i=1}^{n}\left(1-S_{e}\right),\\ F_{i}^{p}=F_{x}^{n}\cdot F_{i}=\sum_{i=1}^{n}\left(1-S_{e}\right), \end{array}$$

where *S*_*i*_ represents the reliability index of the parallel system; *F*_*i*_ represents the reliability index of the hybrid system; and *S*_*e*_ is the reliability of the individual nursing information or the basic information system of a single patient that makes up the parallel system [24]. The nursing system includes units such as outpatient service, registration, and infusion. Each department, such as the nephrology department to be studied in this article, is equivalent to the subsystem in this mathematical model method.

## 3. Experiment Preparation

### 3.1. Research Object

Inclusion criteria of experimental subjects are as follows:

  Step 1: nephrology patients who meet the diagnostic criteria during the recovery period
  Step 2: stable vital signs
  Step 3: patients with cognitive dysfunction who cannot cooperate with the investigator are excluded
  Step 4: nephrology nursing work for more than half a year
  Step 5: pass the annual assessment

### 3.2. Experimental Method

1. This article investigates the patients' satisfaction of the nursing business process in the nephrology department of a third-class hospital in Guangzhou. Through literature research, expert consultation, and interviews, the preparation of the questionnaire was repeatedly revised, and the questionnaire was designed and carried out for the satisfaction of patients in nephrology and related nursing staff, and the reliability and validity of the questionnaire were tested to ensure the validity of the questionnaire. Through the descriptive statistics of the questionnaire and the satisfaction results of medical and nursing integration, a comprehensive evaluation of the construction of information integration is carried out.
2. Using the nursing business process reengineering theory to build a nursing business process model and using genetic algorithms to analyze the model will have a certain effect on the analysis of the role of integrated nursing information construction, medical staff, and nephrology patients' satisfaction.
3. wo experiments were conducted, which are as follows:

  Step 1: expert consultation and interview on information literacy indicators of nursing staff
  Step 2: analysis of the missing items of nursing information in the Department of Nephrology

### 3.3. Experimental Results

The survey results show that 87.5% of patients in the nephrology department are dissatisfied with the current hospital's work efficiency, and 85.7% of the nursing staff in the nephrology department are generally satisfied with the information management of the current department. After the implementation of the hospital's information integration system, patient satisfaction is as high as 98.2%, and the satisfaction of medical staff reached 94.2%. Through the analysis and design of each function in the mobile nursing system based on the Internet of things, the following functions are mainly realized [25]. The nursing staff is not only at the nurse station but can also read the patient's medical orders at any time in the patient's ward or other places in the hospital, and they can also enter physical signs information, dispensing medicine for patients, and other operations [26–30]. It is not necessary to record the physical signs in the book during the rounds and then return to the nurse's station to re-enter them. The handheld mobile terminal PDA can be used to scan and record in real time. The most important thing is to complete other tasks related to medical care.

## 4. Construction of Integrated Nursing Information in Nephrology Department

### 4.1. Feasibility of Constructing Integrated Nursing Information in the Nephrology Department

The introduction of modern computer and communication technology into the medical field has extremely practical value. The integrated nursing information system adopts the operation mode of sending and receiving at the same time. It can ensure that the nursing work is carried out in an orderly manner and that the nursing needs of patients are met. Build a network-based medical care information service platform in a short time and gradually integrate relevant information resources of the hospital. The improvement in business management work is a feature of current research for the research of intelligent nursing path information management systems, which has important economic and social value [31, 32]. In order to study the important value of integrated nursing information more intuitively in the department of nephrology, it has been carried out.  Figure 1 is operational process model diagram of the integrated information system.

The nursing business process model diagram shows that the nursing work is based on the basic information of nephrology patients entered into the hospital database. The patient's medical care information terminal fills in the patient's personal medical record information through the patient's family members and submits medical care online, which shortens the complicated procedures of traditional care and saves manpower and material resources to a large extent. However, the staff is required to classify the patient care information filled out by the patient personnel and then input the data into the computer for data processing [33–35].

Nurses can read or enter patient information through the system at any time, and the computer will generate the dynamic changes of the patient's important physical signs and doctor's orders. While saving manpower, it also avoids the introduction of errors in the transmission and entry process. At the same time, nursing staff can analyze specific problems and flexibly change nursing methods and nursing items so that patient care is more objective and fairer. Nurses can more accurately grasp the doctor's diagnosis and treatment intentions based on computer prompts, and all payment, medicine withdrawal, and dispensing information are entered into the system, reducing communication barriers between departments. In this regard, we compared the work efficiency of nephrology nurses before and after the implementation of integrated information management and recorded the data in Table 1.

According to the comparative analysis of the data compiled in Table 1, it is found that the work efficiency of the nephrology nurses has been greatly improved after the implementation of integrated information management. The background program of the information integration system performs calculations based on the entered patient information data, which saves all kinds of manual time and energy. In general, the waiting time for patients in line for consultation, the time for doctors to diagnose, the filling of cases based on the diagnosis, and the time for medication are all reduced to one-half of the original. This data strongly confirms that the integrated construction of nursing information is the best choice for the current development of hospitals, society, and medical care.

The main function of the system test is to analyze, summarize, and correct the errors of the system in the test so that the functional requirements in the mobile nursing information management can be correctly realized in the system, and the nonfunctional requirements can also be improved. The mature system can better meet people's working habits and make the operation easier.  Figure 2 shows the function test of the nursing information system in the department of nephrology.

### 4.2. Application Analysis of the Integration of Nursing Information in the Nephrology Department

According to the actual operation users of the integrated nursing information system in the overall medical unit, combined with the analysis of the needs of doctors and patients, and combined with various business operations, the specific user roles involved in this research have been determined. They are medical patients and medical staff (this experiment is mainly for nursing staff) and information system managers. This article selects the nephrology department of a third-class hospital in Guangzhou to conduct questionnaire surveys and interviews with patients to study the application of integrated nursing information. The personnel participating in this experiment include the specific user roles in the system, medical patients, medical staff, and system administrators. In the first round of experiment, a questionnaire survey was conducted for medical staff, and the basic statistics of the people who received the questionnaire survey are shown in Table 2.

In the first step of this round of experiment, the 15 questionnaires prepared were distributed to 15 nurses from the clinical nursing department, and they were invited to fill them in truthfully to ensure the authenticity of the experiment. After the subject to be investigated was completed, the content of the questionnaire was evaluated to confirm whether it meets the feasibility standard of this experiment. The evaluation is recorded in Table 3.

In order to follow the principles of goal, science, objectivity, measurability, and simplicity, this questionnaire has a recovery rate of 100% and an effective rate of 100%. The experimental process and experimental results carried out have reference and certain research value.

Information literacy is the foundation of evidence-based nursing and the key standard of nursing information ability. In addition, information literacy can improve the lifelong learning skills of nurses. The information ability of nurses requires nurses to have basic information technology skills and use these information technologies to carry out clinical practice and scientific research to achieve the best nursing practice. According to the search data, 73% of nurses in my country currently choose colleagues when they encounter clinical problems, 89% of nurses have never used the hospital library, 73% of nurses do not use survey reports, and 92% of nurses consider problems when they encounter problems. Some of them use the Internet and the World Wide Web, but more than 80% of this group have never used a database. Due to the knowledge gap in information literacy, the limitation of access to high-quality information resources, and the attitude of not paying attention to research, nursing staff are not fully prepared to provide qualified nursing work. To this end, we conducted statistics on the information literacy of these 15 personnel, and the data is recorded in Figure 3.

The data shows that 15 nursing staff's ability to acquire nursing information is insufficient. Even though they are aware of the importance of nursing information, under the influence of existing conditions, the use of nursing information and the ability to evaluate it after use cannot be exercised. The level of nursing informatization in our country is still at a low level, and the level of information literacy of nursing staff needs to be improved. The integration of nursing information provides powerful conditions, a broad platform for improvement, and unlimited development space to promote nurses to understand the value of information literacy and improve their own information literacy.

In the second round of experiments, in response to the common problems in current nephrology care, such as lack of timely drug supply, insufficient nurse-patient communication, patients not in the ward or uncooperative, or family members interrupted, interviews were conducted with these 15 interviewees. And to sort out and analyze the missing nursing information items in the department of nephrology, the data is sorted in Figure 4.

During the interview, it was learned that nurses often ignore patients' physiological symptoms and psychological symptoms such as anxiety and depression. Nursing assessments such as pain assessment, nutritional assessment, psychosocial assessment, adverse reaction assessment, condition observation, and regular assessment need to be carried out regularly due to work. The amount of work is too large, and the work is too complicated to take care of; when arranging the work flow, life care will be placed at the end, and life care is prone to omissions after the treatment operation is completed; the psychological care and the nursing intervention involved in the nursing intervention during the nursing continuation work the end-of-life care is still not enough. With the integrated nursing information system, various detailed nursing work can be carried out in an orderly and stable manner. This conclusion can be demonstrated in Table 4.

Nursing staff can quickly and accurately record the patient's personal information data, which greatly improves the satisfaction of patients and nursing staff. Integrated information can refine and decompose nursing work, optimize each step from the smallest unit of quality problems, and establish a medical model that can be controlled in real time. This can greatly reduce the working time of nursing staff, rationally arrange the work process, and play a role of supervision. The implementation of the integrated information system platform can seamlessly connect medical treatment, dispensing, basic nursing, and other processes. Nurses and patients can share all the patient's medical treatment information so that the communication between doctors and nurses can be more accurate and timelier. The work process was optimized, the cooperation between medical staff was promoted, the health guidance was further implemented, the quality of nursing service was deepened, and the nurses' enthusiasm for work was aroused.

As the recipient of the nursing work flow and the director of the nursing staff, the patient occupies an important position in the integrated nursing information system. Five inpatients with renal disease in the department of nephrology were selected using statistical methods to participate in this study on the integration of nursing information in the department of nephrology (numbered to protect personal privacy).  Table 5 displays basic statistics of patients.

We talked with these 5 patients. After the information integration system was adopted, they analyzed the nursing work satisfaction evaluation of the nurse staff and solved the problems of the patients' concerns in nursing work after information integration.  Figure 5 presents a comparison of patients' satisfaction with nursing work before and after.  Table 6 displays comparative analysis before and after patients' concerns.

According to data analysis, these five interviewees believe that the construction of an information integration system has had a great effect on the nursing work of nurse staff, and that the staff's work is in place; before the information integration management, there is, for example, the caller fails to receive a response from the nursing staff within 5 minutes, fails to monitor on time according to the doctor's advice, lacks health education, and their physical and psychological care needs are not met. These problems have been properly resolved through the integration of nursing information, which has improved patients' satisfaction with treatment.

## 5. Conclusion

With the development of the social economy and the advancement of medical technology, the medical model centered on diseases in the past is far from being able to meet the medical needs of current patients. The medical model of “bio-psychosocial” centered on patients is more suitable for current medical care. Serving patients and effectively solving the problems encountered by patients in the process of hospital visits is the purpose of the development of an integrated nursing information system, and it is also its primary task. While the system can conveniently display relevant information about patients' visits and hospitalizations, it can also collect detailed patient clinical data information and provide medical staff with the right to retrieve and check patient-related information without being restricted by time and place, so that it can be used by the medical industry. Scientific research, health care, and medical levels provide effective diagnosis and treatment information. The current situation we are facing is a very complex situation with various heterogeneous data and different application systems. The lack of unified planning, unified interface standards, and a unified data storage platform will cause overlap of various functions and duplication of nursing business processes. The integrated information platform is based on the existing information system and established in accordance with the requirements of joint integrated operations. The knowledge and management methods of the medical system can be enhanced through the clinical information management system in the ward. Improving in business management is a feature of current research for the study of integrated nursing information management systems, which has important economic and social value.

## Figures and Tables

**Figure 1:** Operational process model diagram of the integrated information system.

**Figure 2:** Function test of the nursing information system in the department of nephrology.

**Figure 3:** Nursing information literacy indicators for consulting and interviewing nurses.

**Figure 4:** Nurses' perception of lack of nursing work.

**Figure 5:** Comparison of patients' satisfaction with nursing work before and after.

**Table 1:** Comparison table of medical and nursing work efficiency before and after the implementation of information integration management (minutes).

Time	Queuing time	Diagnosis time	Dispensing time	Time to take medicine	Payment time
Before implementation	10–15 minutes	7–10 minutes	2–3 minutes	10–12 minutes	3–5 minutes
After implementation	6–8 minutes	5–7 minutes	1–2 minutes	6–9 minutes	2–3 minutes

**Table 2:** The basic situation of the personnel participating in the experiment.

Number of people	Gender	Age	Working time	Field of work
10	Female	22–35	1–7 years	Clinical nursing
5	Male	22–27	Half a year–4 years	Clinical nursing

**Table 3:** Questionnaire recovery.

Number of investigation rounds	Distribute the questionnaire	Recycle the questionnaire	Valid questionnaire	Recovery rate (%)	Efficiency (%)
First round	15	15	15	100	100
Second	15	15	15	100	100

**Table 4:** Nursing work business evaluation and improvement table.

Project	Before information integration	After information integration
Competency assessment for nurses	85.7%	94.2%
File recording time (h)	1.5–2	0.5
Record pass rate	91.3%	97.9%
Patient satisfaction	87.5%	98.2%
System satisfaction	89.1%	98.9%

**Table 5:** Basic statistics of patients.

Numbering	Age	Gender	Type of disease	Length of hospital stay
A	43	Male	Acute renal pelvis	Two weeks
B	45	Female	Nephrotic syndrome	One month
C	29	Male	Nephrotic syndrome	One month
D	36	Male	Chronic renal failure	Over one month
E	42	Male	Acute renal pelvis	15 days

**Table 6:** Comparative analysis before and after patients' concerns.

Problems	Before	After
The pager did not respond within five minutes	Not effectively processed	Troubles solved
Monitor on time according to doctor's advice	Slightly dealt with but not enough	Resolved and satisfied
Health education during hospitalization	Not effectively processed	Troubles solved
Pain care for patients with kidney disease	Not effectively processed	Resolved and satisfied
Psychological care for patients and their families	Slightly dealt with but not enough	Troubles solved

## Data Availability

The simulation experiment data used to support the findings of this study are available from the corresponding author upon reasonable request.
